RETRACTED

# Influence of Knowledge-Based Employee Incentive Construction on Innovation Performance Using Psychological Capital

**DOI:** 10.1155/2022/9424068

**Published:** 2022-09-09

**Authors:** Yuanqin Ge, Yang He, Zhen Huang, Xiaomeng Sun

**Affiliations:** ^1^School of Economics and Management, Shihezi University, Shihezi, Xinjiang, China; ^2^Normal College, Shihezi University, Shihezi, Xinjiang, China

## Abstract

**Background:**

Driven by the Silk Road Economic Belt idea, Xinjiang Uygur Autonomous Region can fully play its regional advantages and innovate the open economic system. It can transform and upgrade industrial structures with strong regional characteristics and advantages in Shihezi.

**Objective:**

The purpose is to explore the impact of knowledge-based employee incentive mechanism (EIM) on innovation performance. It is hoped to innovate the knowledge-based worker (KBW) management in Shihezi enterprises.

**Methods:**

Based on the psychological theory, the actual production, and living conditions in Shihezi, a questionnaire survey is conducted on the KBWs of typical enterprises in Shihezi. The questionnaire is designed by considering the characteristics of KBWs in Shihezi City under the Development Strategy of Western Chinese Cities. In addition, relevant structural equation models and hypotheses are proposed to comprehensively explain the relationship between psychological capital (PsyCap), EIM, and employee innovation performance (EIP).

**Results:**

Among the KBWs of Shihezi enterprises surveyed, the proportion of male and female employees is basically balanced, and both groups have bachelor's degrees or above. They are mostly young, with a relatively short working year. Most employees are in the rising stage of career development. The overall scores of KBWs on the PsyCap, EWM, and EIP scales are all above 3.5, a high overall score. Model analysis and hypothesis verification show that Shihezi knowledge-based EIM significantly affects EIP and PsyCap. The PsyCap has a positive impact on EIP. The KBWs' PsyCap plays an intermediary role in EIP.

**Conclusion:**

The research results provide an objective reference for Shihezi enterprises to improve the innovation performance of KBWs. It enriches the theoretical research of Shihezi enterprise innovation and provides a theoretical basis to improve collaborative innovation performance.

## 1. Introduction

A new round of global scientific and technological revolution and industrial reform is accelerating, and scientific exploration is expanding from the micro to the full-scale universe. The collective intelligence and green technological revolution will trigger a major adjustment of the international industrial division. Disruptive technologies continue to emerge, such as human-computer interaction (HCI) technology in artificial intelligence (AI) [1–3]. Meanwhile, institutional, management, business model, industrial, and cultural innovation are becoming the core strategies for many countries, including China, to seek a competitive advantage. In China, the 18th CPC National Congress proposed implementing the innovation-driven development strategy. It emphasized that scientific and technological innovation is the strategic support for improving social productivity and comprehensive national strength. Modern enterprises can only face various challenges by investing in continuous innovation and development [4]. Innovation is directly related to an enterprise's competitive advantage and sustainable growth [5]. Technological innovation strategy is the basic principle to improve the innovation performance of knowledge-based workers (KBWs). Under this background, the demand of enterprises for knowledge-based workers is gradually increasing. KBWs generally have high academic qualifications and strong working abilities. Most of them are engaged in mental work, which is an important force for the innovation and development of enterprises [6].

RETRACTED

Enterprise development has also brought challenges. For example, KBWs in Xinjiang also face many difficulties with intensified enterprise competition, bearing more work pressure than ever before. These pressures have adversely affected employees' lives and work, reducing work efficiency and leading to resignation. The local enterprises complain about the impact of these difficulties on employees' personal development and enterprise stability [7]. Therefore, the psychological situation of KBWs must be attended to during enterprise development, and scientific incentives should be devised to promote employee innovation performance (EIP). Psychological capital (PsyCap) deals with the psychological state of individuals. It explains EIP and is considered the key determinant of the future organizational competitive advantage and the true valuable asset of the enterprise [8]. Accordingly, this work analyzes the influence of knowledge-based employee incentive mechanism (EIM) on EIP from the perspective of PsyCap.

Shihezi, in the border area of northwestern China, has a distinct economic and social development from inland cities. With the orderly advancement of China's Great Western Development Strategy and the Belt and Road Initiative (BRI) in recent years, the development of all sectors of society in Shihezi has ushered in tremendous changes [9]. Shihezi has seen a decade of economic boom. Various ownership economies have become influential carriers for Shihezi to fully open up to the outside world and build a regional international trade center. This is vital for expanding the scope of international trade, increasing employment rates, and increasing taxation [10]. At the current stage, Shihezi strives to expand the world market, deepen exchanges and cooperation with various countries and regions, and develop an open economy. Shihezi has become an essential force in building the Silk Road Economic Belt [11]. President Xi stated at the 3rd Xinjiang Work Symposium of the CPC Central Committee that Xinjiang should fully play its regional advantages. It should innovate the open economic system to strengthen, optimize, and upgrade industrial development and structures. In this context, the demand for KBWs in Xinjiang is more urgent than ever before. At the same time, Shihezi's KBWs also have some difficulties. Unlike the rest of China, Shihezi enterprise has unique characteristics in training KBWs mainly due to the geographical environment. For example, employees need more external incentives to enhance internal incentives and PscyCap and reduce turnover intention. Therefore, scientific management methods can improve the Shihezi KBW's EIP and promote the development of Shihezi enterprises and society according to the policies of Xinjiang.

RETRACTED

According to the concepts of psychology and management, KBWs in border areas are sampled. The PsyCap of employees and the influence of EIM on EIP are explored, considering the actual situation in Shihezi. Based on previous research, the relationships among the three variables of employees' PsyCap, EIM, and EIP are investigated through case analysis. It is hoped to provide a practical reference for enterprises to improve the innovation performance of employees.

## 2. Literature Review

### 2.1. Connotation Analysis of Relevant Concepts

PsyCap is generally considered to be a positive psychological state shown by an individual during growth and development. It is an organic combination of an individual's self, social relationships, professional development, moral concepts, life goals, and beliefs [12]. Studies have shown that PsyCap was influential in promoting individual growth and performance improvement. Effectively evaluating and measuring PsyCap has always been a key concern. Regarding work, the influencing factors of enterprise employees' PsyCap include three principal elements: individual, environmental, and leadership. Individual elements refer to factors about personal traits, personality, and basic situations, such as age, gender, educational background, initiative, self-emotion, self-evaluation, psychological safety, and self-esteem [13]. Environmental elements are the surrounding environment and the organization's influence, including the organizational atmosphere, organizational culture, and working conditions. The leadership elements include leadership behavior and ability [14]. PsyCap helps employees maintain optimism, gain confidence, and outlook for the future and show others' gratitude and high emotional intelligence. Thereby, PsyCap contributes to employees' personal growth and the entire enterprise's good development [15].

RETRACTED

Innovation performance is an essential indicator that describes the innovation achievements of enterprises. In the meantime, innovation performance is also a core component of employees' performance and plays a key role in providing enterprises with sustained competitive advantages [16]. Innovation is a vital factor for the stable development of an enterprise. Enterprises with less innovative employees will lose their competitive advantage. In particular, EIP refers to the innovative activities of employees during work and the perceived measurable results that benefit the enterprise. These include the ability to put forward innovative ideas, apply new methods, utilize new technologies, and summarize work tips [17, 18]. They also include innovative activities-induced outcomes [19], applications, and effects [20]. The EIP can be measured by innovation input, output, and process or comprehensive measurement [21] with five indicators: success rate, time, investment return rate, fulfillment, and results. In general, the influencing factors of innovation performance can be divided from the organizational or the individual perspectives. Organizational incentives, organizational climate, leadership style, and organizational learning ability will influence innovation performance [22]. From an individual perspective, employees' happiness, job satisfaction, emotional intelligence, and good interpersonal relationships can all impact innovation performance.

Employee incentive is the psychological process of continuously stimulating individuals through internal or external stimuli to maintain an excited state [23]. According to management analysis, incentives can be based on content, process, or comprehensive factors. Content-based incentive discusses the essential pursuit of individuals. Process-based incentive studies how people are motivated to take action; it believes that there is a necessary connection between behavior and employees' expected needs. Comprehensive incentive involves many aspects, such as incentives' starting point and process. It controls the relevant variables and considers comprehensive factors, such as reward content, system, organizational division of labor, goal setting, and fair assessment [24].

RETRACTED

KBWs possess some knowledge, symbols, or concepts and use the information they have for work. With the development of society and the diversified labor divisions, the definition of KBW is also being extended. KBWs have the following three basic elements: (1) they can master knowledge or skills and use them proficiently in work; (2) they have strong learning and innovation ability and can integrate relevant resources for innovative research in their work; and (3) they use the learned knowledge to bring benefits and value to the organization [25]. Additionally, KBWs also have higher academic qualifications. They pursue self-worthiness, dare to try new and challenging problems, are highly independent, and value spiritual encouragement and recognition. In other words, they value the spiritual rewards at work over external rewards. These talents are often engaged in mental works, with a relatively free working environment and time schedules. Notably, the work of KBWs is difficult to quantify since all team members have shown contributions.

### 2.2. Literature Review of Relevant Research

#### 2.2.1. Research on Employees' PsyCap

Definitions of PsyCap are inclusive. Youssef-Morgan [26] believed that PsyCap manifested an optimistic and cheerful mood, self-confidence, hopefulness, and faithfulness. Luthans and Youssef-Morgan [27] concluded that hope, efficiency, resilience, optimism, and inner hope were the principal factors that constituted PsyCap. Luthans et al. [28] explained that PsyCap and employees' internal attitudes, external behaviors, and performance results had significant relationships. The individual's PsyCap could be affected by external effects.

The influencing factors of PsyCap and their impact on job performance are also the focus of researchers. Paek et al. [29] surveyed employees of 15 five-star hotels in South Korea. The results showed that work involvement affected PsyCap. Frontline employees with higher PsyCap were involved in work and likely to show job satisfaction and emotional investment in the organization. Manzano-Garcí and Ayala [30] proposed that PsyCap significantly impacted mental health and that PsyCap reduced employees' job burnout, further improving work efficiency. In short, the impact of PsyCap on the development of enterprises and organizations is substantial. PsyCap is directly related to employees' job performance and will affect enterprise development.

#### 2.2.2. Research on EIP

EIP can be explained from multiple dimensions. Abbas and Raja [31] considered that innovation performance included the innovation of employees in the work process and the results obtained by innovations. Rylková and Chobotová [32] divided innovation into three levels. An enterprise's permanent and overall innovation management integrated all strategic tasks, such as implementing new projects and innovation management activities. The input and output of special projects transformed innovative ideas into products. The future development of innovative products was also studied. Mardani et al. [33] researched the innovation performance of 120 enterprises in Iran. The results showed that knowledge management activities could directly affect innovation and organizational performance and indirectly improve innovation capabilities. Raja et al. [34] revealed a positive correlation between quality practices and enterprises' innovation performance. Moreover, factors such as business environment uncertainty, enterprise size, financial resources, and corporate culture could all affect this relationship.

RETRACTED

At this stage, the development of KBWs in Shihezi has achieved remarkable results. The distribution of KBWs in various industries is becoming reasonable and scientific. All kinds of talents have been transferred to key economic and social construction areas in an orderly manner, and the scale of KBWs in the secondary and tertiary industries has continued to expand. At the same time, the talent quality has been gradually improved, and the training scale has been expanded. Shihezi local government actively develops key fields and industrial positioning, adjusts talent introduction ideas, innovates talent introduction methods, and constantly introduces innovative, high-level, urgently needed, skilled, and practical talents. With the support of policies, the environment for talent development is also optimized. The investment in talents has increased year by year, and the incentive and guarantee mechanism for talent distribution has been improved. The scientific and legal level of talent management has been significantly improved. Shihezi's talent plan has been implemented and accelerated. The importance of introducing scarce professionals and local training talents has been emphasized. Grassroots KBWs and talents in short supply are cultivated purposefully for social development. KBWs are the main factor of social innovation. Therefore, improving the innovation performance of KBWs plays a vital role in promoting social and economic development.

#### 2.2.3. Effect of Knowledge-Based Employee Incentive Mechanism (EIM)

The method and effect of EIM have always been the key to business management. Besides, as the KBW becomes prominent in enterprise innovation, research on the effect of knowledge-based EIM has attracted widespread attention worldwide. The results of Wang and Tsai [35] on 586 questionnaires on leaders showed a one-way direct positive impact between resources, management practices, organizational incentives, and organizational innovation. Internal incentives directly affect the creativity of employees. Bryson and Freeman [36] argued that employees could be motivated through stock purchase plans. Their results showed that this method could further improve the production efficiency of employees and the loyalty of employees to the enterprises. Sung et al. [37] collected data from 227 enterprises in South Korea and revealed that salary incentives could improve employees' workability and work attitude, thereby improving the enterprise's operations and financial performance. Han et al. [38] studied the relationship between human resource practice management and innovation by introducing authorized leadership as a boundary condition in the analysis framework. They discussed the regulatory role of authorized leadership on human resource management practice and team knowledge sharing through empirical analysis. The research results demonstrated the substitution of human resource management practice and authorized leadership in knowledge-intensive teams. Zhao et al. [39] examined the relationship between employees' leadership, professional and organizational identity, and applied leadership behavior and social identity theory. The results showed that leadership behavior and social identity theory significantly impacted the mechanism of EIP. Singh et al. [40] studied the relationship between human resource management practice and innovation performance. The structural equation model (SEM) analyzed the collected data to check the research assumptions. The results showed that knowledge sharing could adjust the impact of social capital on innovation performance. To sum up, employee motivation can often positively affect enterprises and companies. The above literature does not explain the specific content of employee incentives in detail, which is also the main deficiency and the research gap that needs to be filled. This work studies how to scientifically analyze the specific content of employee incentives in practical application to promote the common development of employees and enterprises.

RETRACTED

## 3. Research Methodology

### 3.1. Profile Analysis of KBWs in Shihezi

With the continuous and effective promotion of China's Western Region Development Strategy and the BRI, Shihezi's socioeconomic scale and gross domestic product (GDP) have significantly increased. In this context, all sectors of Shihezi society have turned their attention to KBWs. Shihezi's colleges and universities, corps, enterprises, and institutions have launched a series of talent attraction measures to absorb more knowledge-based talents. Through policy support and the impact on the overall environment, Shihezi enterprises have flourished, and the comprehensive strength and overall business environment have been effectively improved. The successful implementation of the talent introduction project has attracted outstanding talents worldwide, improved the EIM, and expanded the KBWs of the Shihezi enterprise.

### 3.2. Questionnaire Design

KBWs generally work in high-tech enterprises or emerging industries with certain patents. Here, employees of high-tech enterprises or emerging industries in Shihezi are surveyed to extend the sample range. The samples are employees of three enterprises in Shihezi: *X* enterprise engaged in textile, B enterprise engaged in food processing, and *T* enterprise in the chemical industry. Overall, 300 questionnaires are distributed, recovering 280 valid ones, with a recovery rate of 93%.

The three variables involved are PsyCap, EIM, and EIP. The PsyCap measurement questionnaire refers to the PsyCap scale developed by Hou et al. The original scale includes 4 dimensions and 49 questions involving task-based PsyCap associated with completing work tasks, relational PsyCap associated with peripheral relationship processing, learning PsyCap associated with knowledge learning, and the innovative PsyCap. Regarding the actual situation in Shihezi, two dimensions of task-based PsyCap and innovative PsyCap in the scale are selected, totaling 8 questions. The innovation performance scale developed by Yao and Heng [41] is adopted with two dimensions: innovation action and innovation effect. The questions are properly integrated based on the original dimension of the scale. The innovation action and innovation effect each include four questions, totaling 8 questions. The EIM scale includes 15 questions analyzed from four dimensions: corporate welfare, employee salary, employee promotion path, and corporate culture. All questions are based on the 5-point Likert item, in which 1 point to 5 points, respectively, represent “strongly disagree” to “strongly agree.” The higher the score, the higher the relevant measurement level.

### 3.3. Research Hypothesis and Model Establishment

Based on the above theoretical data, the following hypotheses are put forward:

  H1: Knowledge-based EIM influences EIP significantly and positively
  H2: Knowledge-based EIM influences employees' PsyCap significantly and positively
  H3: PsyCap influences EIP significantly and positively
  H4: PsyCap plays a mediating role between EIP and EIM

At the same time, based on the above hypotheses, the research model of the relationships among knowledge-based employees' PsyCap, EIM, and EIP is shown in Figure 1.

RETRACTED

## 4. Results and Discussions

### 4.1. Profile Analysis of Research Samples

First, the basic situation of the research samples is analyzed, including the statistical analysis of gender, education, working years, and age. The results are summarized in Figure 2.

As shown in Figure 2, the proportion of men and women in the research samples is basically balanced. Among the 280 surveyed employees, 157 are men, accounting for 56.07%; 123 are women, accounting for 43.93%. As for the distribution of academic qualifications, KBWs generally have a bachelor's degree or above. There are 95 graduates and 12 doctoral students, indicating that the KBW in Shihezi has a high educational background. The statistics for working years show that more than half of employees have worked for less than 3 years. Employees working 1–3 years account for the majority. At the same time, most employees are young people under 35.

Statistical analysis is performed on the results of the questionnaire survey. The results of the PsyCap, EIP, and EIM are shown in Figures 3(a)–3(c), respectively.

As shown in Figure 3, in the PsyCap scale, the task-based PsyCap dimension has an average score of 3.87 points and a standard deviation (SD) of 0.732. The innovative PsyCap dimension has an average score of 3.56 points and an SD of 0.915. In the EIP scale, the average score of the innovation action dimension is 3.68 points, with an SD of 0.869; the average score of the innovation effect dimension is 4.01 points, with an SD of 0.766. In the EIM scale, the average scores of corporate welfare, employee salary, employee promotion path, and corporate culture are 3.89, 3.53, 3.57, and 3.94, respectively, with SDs of 0.804, 0.791, 0.941, and 0.779, respectively.

The above results show that KBWs in Shihezi have high scores on the PsyCap, EIP, and EIM, with scores above 3.5 in all dimensions. The score of the innovation effect is 4.01, ranking the highest, while that of the employee salary is 3.53, ranking the lowest.

### 4.2. Reliability and Validity Analysis of the Questionnaire

The reliability and validity of the survey results are analyzed using the SPSS21.0 software. In the category of reliability analysis, the CITC value and Cronbach's *α* coefficient are considered. The PsyCap scale is set to *Q*1; the EIP scale is set to *Q*2; and the EIM scale is set to *Q*3. Besides, each question in the scale is labeled in turn. The specific scores of the three scales are shown in Figures 4(a)–4(c).

The CITC value is generally required to be greater than 0.5, and Cronbach's *α* coefficient value is greater than 0.7. As shown in Figure 4, each question in the scale meets the above requirements. Furthermore, Cronbach's *α* coefficient of each dimension is greater than 0.8, indicating that the scale's reliability is very good, meeting the reliability requirements.

RETRACTED

The scale's validity is tested through the Kaiser–Meyer–Olkin (KMO) and Bartlett sphere tests. The results are provided in Table 1.

Table 1 reveals that the KMO values of PsyCap, EIP, and EIM scales are 0.921, 0.905, and 0.934, respectively, which are all greater than 0.9. The Bartlett sphere test observations are 5,492.937, 3,021.347, and 2,084.548, all greater than 0.9. Moreover, all the *P* values are 0.000, less than the given significance level of 0.01, indicating a correlation between the variables. Hence, the scale has passed the validity test.

### 4.3. Correlation Analysis of Various Variables

The variables' dimensions undergo correlation analysis, and the results are summarized in Table 2.

Table 2 suggests that the correlation coefficients of the various dimensions of the variables involved are all less than 0.8, without severe collinear problems. Therefore, all dimensions of the three variables are significantly correlated.

### 4.4. Verification of Research Hypotheses

A structural equation model is constructed referring to Giorgi's approach [42]. The AMOS21 software is applied to fit and analyze the model. First, the overall theoretical model is examined. The absolute fit, the incremental fit, and the reduced fit are considered to fully analyze the model. The results obtained are shown in Figure 5.

As shown in Figure 5, *χ*^2^/df = 2.230, indicating that the model fits well. The GFI value is 0.958, which meets the expected requirements. The RMSEA value is 0.802, which indicates a moderate fit. The values of CFI, NFI, TLI, and IFI are all greater than 0.8, indicating that the model fits well. The values of PGF, IPNF, and IPCFI are all greater than 0.5, indicating that the model has achieved the expected ideal standard. In summary, the model's absolute, incremental, and reduced fit are all within the acceptable range. Thus, the model fits well. At the same time, the principal effects test is performed; that is, the relationship between the independent and dependent variables is tested when the mediating variable is not added to the model. In other words, the influence of EIM on EIP is explored. The specific results are as follows:

According to data in Table 3, the knowledge-based EIM can promote EIP. Thus, hypothesis 1 holds.

After the mediating model is added, the overall test is performed. The specific results are summarized in Table 4.

RETRACTED

As shown in Table 4, in the second path, the estimate is 0.847, and *P* < 0.001, indicating that EIM has a significant positive impact on PsyCap. Hence, hypothesis 2 holds. In the third path, the estimate is 0.886, *P* < 0.01, indicating that PsyCap has a significant positive impact on EIP. Therefore, hypothesis 3 is established. Moreover, the corresponding coefficient is found to decrease in this model, indicating that PsyCap plays a mediating role; that is, hypothesis 4 is valid.

## 5. Conclusion

The KBW of different enterprises in Shihezi is sampled by considering their basic situations, and relevant models and hypotheses are proposed to investigate the relationships among PsyCap, EIP, and EIM. The key conclusions are as follows. The proportion of men and women in KBWs of Shihezi enterprises is basically balanced, which are 56.07% and 43.93%, respectively. KBWs generally have high academic qualifications, with a bachelor's degree or above. Most KBWs are young and in the career development stage. The KBWs in Shihezi enterprises have scored high on the three scales of PsyCap, EIP, and EIM. The EIP is the highest, with 4.01 points. Moreover, the research scales have passed the reliability and validity tests. The model and relevant hypotheses are proposed. Testing and verification reveal that the model fits well and meets the expected standard, and the research hypotheses hold. Compared with previous research, the proposed model fully integrates the basic situation of Shihezi. A targeted survey of enterprises in Shihezi is conducted. In view of the research limitations, which used cross-sectional data, future studies can use multitemporal longitudinal studies to reduce endogeneity problems. Besides, the enterprises in different industries are investigated to generalize the survey results and make the survey more practical [43]. The results have strong pertinence, focusing on developing enterprises in Shihezi. The findings have excellent practical application values.

This research provides the following clues to the innovative development of Shihezi enterprises. (1) Talents guarantee enterprise innovation. Therefore, supplementing and cultivating talents must be carried out in Shihezi enterprises. For this reason, collaborative innovation in Shihezi enterprises must change the employment strategy to cultivate KBWs with a comprehensive and reasonable view, construct cultural ideas, and encourage open management. Meanwhile, they should actively cultivate leaders in collaborative innovation projects, encourage employees to refine themselves, and offer platforms for employees to innovate. (2) Because of the geological conditions, Shihezi enterprises should improve employee salaries and education for their children to attract more KBWs. Favorable policies must be followed to enhance KBWs' PsyCap, allowing them more extensive development. The main contribution is to provide a theoretical basis for the performance innovation of Shihezi enterprises. In addition, the research has certain limitations. The potential limitation lies in the insufficient consideration of employees' psychological factors in modeling the performance evaluation and talent attraction mechanisms. The theoretical research results of Shihezi KBWs as innovation subjects are relatively few from the current research field of employee and enterprise innovation. Improving employees' professional skills and reducing ineffective activities can further improve the innovation performance of enterprises. Examining the EIP factors can enrich the research on Shihezi enterprise innovation. It is expected to provide a theoretical basis for improving Shihezi enterprise collaborative innovation performance.

RETRACTED

## Figures and Tables

**Figure 1:** The influence model of PsyCap, EIM, and EIP.

**Figure 2:** Basic statistics of research samples.

**Figure 3:** Analysis of the scale survey results.

**Figure 4:** The CITC value of the scale and the statistical results of Cronbach's *α* coefficient.

**Figure 5:** Evaluation indicator of overall fitness of the structural equation model.

**Table 1:** KMO of the scale and Bartlett test results.

Scale	KMO	Bartlett test	*P*
PsyCap	0.921	5,492.937	0.000
EIP	0.905	3,021.347	0.000
EIM	0.934	2,084.548	0.000

**Table 2:** Correlation between various dimensions.

	Task-based PsyCap	Innovative PsyCap	Innovative action	Innovation effect	Corporate welfare	Employee salary	Employee promotion path	Corporate culture
Task-based PsyCap	1							

Innovative PsyCap	0.768^*∗∗*^	1						

Innovative action	0.594^*∗∗*^	0.546^*∗∗*^	1					

Innovation effect	0.634^*∗∗*^	0.745^*∗∗*^	0.784^*∗∗*^	1				

Corporate welfare	0.715^*∗∗*^	0.760^*∗∗*^	0.732^*∗∗*^	0.799^*∗∗*^	1			

Employee salary	0.613^*∗∗*^	0.784^*∗∗*^	0.702^*∗∗*^	0.702^*∗∗*^	0.750^*∗∗*^	1		

Employee promotion path	0.731^*∗∗*^	0.721^*∗∗*^	0.747^*∗∗*^	0.735^*∗∗*^	0.713^*∗∗*^	0.737^*∗∗*^	1	

Corporate culture	0.714^*∗∗*^	0.765^*∗∗*^	0.729^*∗∗*^	0.799^*∗∗*^	0.786^*∗∗*^	0.762^*∗∗*^	0.786^*∗∗*^	1

Note: ^*∗∗*^*P* < 0.01.

**Table 3:** Regression coefficients of the principal effect path.

Parameter	Value
Estimate	1.032
SE.	0.56
CR.	19.434
*P*	<0.001

**Table 4:** Regression coefficients of the overall model path.

Path	Parameter	Value
EIM ⟶ EIP	Estimate	0.847
	SE.	0.774
	CR.	11.384
	*P*	<0.001

EIM ⟶ PsyCap	Estimate	0.886
	SE.	0.611
	CR.	15.641
	*P*	<0.001

PsyCap ⟶ EIP	Estimate	0.531
	SE.	0.720
	CR.	4.538
	*P*	<0.01

RETRACTED

## Data Availability

The data set can be obtained from the corresponding author upon request.
